The article "Stability and Phase Response Analysis of Optimum Reduced-Order IIR Filter Designs for ECG R-Peak Detection" was published in 2022. Journal: J Healthc Eng.

# Stability and Phase Response Analysis of Optimum Reduced-Order IIR Filter Designs for ECG R-Peak Detection

**DOI:** 10.1155/2022/9899899

**Published:** 2022-04-11

**Authors:** Hemant Amhia, A. K. Wadhwani

**Affiliations:** Electrical Engineering, M.I.T.S, Gwalior, M.P., India

## Abstract

Cardiovascular health and training success can be assessed using electrocardiogram (ECG) data. For over a quarter of a century, an individual's resting heart rate is varying more. As a result, it has become the subject of inquiry and reveals the intricate relationship between the human body and its environment. The autonomic nervous system has impact on blood flow system based on the rate of heartbeats. However, heart rate variation (HRV) characteristics analysis throughout the time period has lack of physical activity information. In the presence of patient movement, ECG signal is suffering from hard artefacts. Time-varying HRV parameters can be derived from low-frequency (LF) and high-frequency (HF) domains of the correct frequency. However, sometimes it is critical to ensuring accurate detection of the R-peak position. The proposed ROIIR (reduced-order IIR) offers 8.8% improvement in peak-to-peak swing than earlier IIR filter. We present an advanced filtering algorithm that is used for R-peak detection.

## 1. Introduction

An individual's heart is a muscular structure that pumps blood through the circulatory system, allowing them to live. If the heart fails, a person will die. Heart illness is the foremost basis of death amongst humans today. Many people die as a result of heart illness. An electrocardiogram (ECG) is a recording of the physical explanation of electrical performance during the heart sequence. In order to discover heartbeat problems, ECG is utilized to assess heartbeat's rate and rhythm. Heart issues can be diagnosed early if they can be monitored by an ECG. Electrocardiogram (ECG) signal is a graphical depiction of cardiac commotion that can be used to identify heart illness.

Various waves, segments, and limited interludes make up the ECG signal. P, Q, R, S, and T are the five basic ECG waves. Information about cardiac disease can be gleaned from P-QRS-T wave patterns and the time interludes amongst crests. The QRS complex, the P and T waves, the QRS-Q wave, the R wave, and the S wave are all critical components in the ECG signal analysis [1]. Humanoid stress, crusade, ECG machine cable dislodgment, machine issue, and lead misplacement can all modify the electrode skin impedance, resulting in a noisy signal that can be hard for computer processing and difficult for a cardiologist to understand. The ECG data must therefore be filtered in order to detect and further process the heartbeat peak. Baseline drifts, power line interference, and ECG noise all contribute to ECG signal noise. Power line interference occurs at medium frequencies, and electromyography occurs at high frequencies; hence, baseline wander is a low-frequency filtering phenomenon. Filters are applied to eradicate these noises. When the noise in the ECG input signal is reduced using filters, the desired information can be extracted [2]. High-pass, low-pass, band-pass, band-stop, and all-pass filters are all used in ECG filtering. Filtering is based on the cut-off frequency; if we lower the cut-off frequency, then lowering the frequency will be allowed to pass through. The low and high frequencies are reduced by a band-stop filter, whereas the high and low frequencies are not affected by an all-pass filter. Filters are divided into two types: analogue and digital. Finite impulse response (FIR) filters and infinite impulse response (IIR) filters are once again two types of digital filters. FIR filters are outperformed by IIR filters in terms of speed and memory requirements. The IIR filter is a recursive filter centred on a sole linear filter, with the current output linked to the preceding input and output. There are less design parameters, less memory needs, and less computational complication in IIR digital filters compared with FIR digital filters [3]. Designing and implementing IIR filters are more versatile since there are fewer limitations. When compared with FIR filters, IIR filters have a smaller number of parameters but are more vulnerable to noise and have a shorter response time. From the analogue filter, a bilinear transformation is used to create the digital IIR filter. Digital filters with a limitless impulse retort are known as IIR filters.

Heart rate variability (HRV), or the temporal deviation between heartbeats, has been increasingly noteworthy in recent years. The precise identification of R-peaks and RR-intervals for physiological interpretation has become increasingly important [1]. Following the transfer of RR interludes into frequency domain moreover in certain frequency bands is known to be associated with activation of the sympathetic and parasympathetic nervous system and central nervous system [1]. Many motion artefacts, such as random or stochastic noise, cause the ECG to deform and the signal-to-noise ratio (SNR) to plummet, especially during physical activity [4–6]. ECG algorithms used in clinical practice are not intended for this determination and so demonstrate high false alarm degrees, resulting in inaccurate HRV measurements. In order to deal with motion artefacts, a number of filter approaches have been proposed. Finite impulse response (FIR) filters are commonly used in many algorithms. It is possible to obtain an undistorted ECG signal from this method because the FIR filter is combined with a delay that is equal to the essential numeral of the filter. A large number of filter coefficients are required by FIR filters to achieve the desired signal characteristics, resulting in a significant rise in the computational burden. Mobile applications, especially those that demand low battery consumption, limit the computer resources available; therefore, computational costs become increasingly significant. Because the FIR filter is bidirectional, we recommend employing a bidirectional infinite impulse response (IIR) filter. It is possible to achieve a great quality output with less filter constants and less computation time using the recursive IIR filter. The problem of familiarizing a phase shift can be avoided by smearing the filter bidirectional [7, 8]. Following the filtering step, we add an R-peak detector founded on an improved methodology to perceive R-peaks to overcome motion artefacts [9]. Extra plausibility checks are needed to evaluate whether the observed event is part of a genuine R-peak or an artefact. In the particular instance of mobile data, R-peak detection rates can be enhanced using these innovations.

## 2. ECG Dataset Details

A total of 18 ECG data were used to contrivance this investigation in the MATLAB surroundings. Each recording lasts for 30 minutes and 5556 seconds, but the time displayed below has been adjusted down to the next second to account for rounding errors. The heart rate is recorded in beats per minute across three R-R intervals [10]. Moreover, same database was applied in one of another research [11].

## 3. Existing Methodology

In research work [12], high-power noise in the ECG was reduced using an IIR Butterworth filter. This claim is backed up by the results of an IIR Butterworth low-pass filter, which demonstrate that the power of the filter signal is lower than that for the noise signal. Li et al. [6] developed an upgraded numeral coefficient IIR filter and associated with straight approaches of numeral coefficient. Low- and high-pass filters created by IIR can reduce both power frequency interference and baseline drift [13].

The Butterworth low-pass filter has a cut-off frequency of 100 Hz, which is used by Gaikwad and Chavan [14] to reduce noise from the ECG data. The result shows a reduction in noise of −18 dB. To eradicate power line noise from ECG signals, the discrete Fourier transform founded algorithm, IIR, FIR, Kalman wavelet, and in addition, advanced-order statistical filtering techniques were applied by Amiri et al. [15]. It has been determined that FIR filtering and IIR filtering improve SNR the most. Elliptic filtering and Butterworth Chebyshev type I, type II, and elliptic filtering were applied by Bhogeshwar and colleagues [16] to reduce noise from ECG signals. Once these algorithms applied to the MIT-BIH ECG database signals, the IIR elliptic filter is said to have increased SNR performance [17].

High-frequency disturbances whose order was experimentally selected were removed by Dhar et al. [17] using a Butterworth low-pass filter. To make the ECG file smaller, we compress the filtered signal using a stringent lossless approach. Das and Chakraborty [7] attempted to sifter ECG indications using FIR and IIR filters. Elliptic filter and Chebyshev type I IIR filters had the highest SNR values in 2 to 4 filter ranges, according to the results. If the filter order is amongst 12 and 14, then the SNR for Chebyshev type II is great [8, 18]. SNR fluctuations in the filter order have been discovered to lead to the selection of the correct filter for ECG filtering. Wavelet transforms can be combined with evolutionary algorithms for enhanced noise removal, according to Ref. [19, 20]. There are 10 ECG signals that were taken from the MIT-BIH arrhythmia record. A low-pass filter was designed by Saini et al. using IIR filters, for example, Butterworth, elliptic, and Chebyshev filters to reduce the electromyography noise [21]. In addition, FIR digital sifters are applied. Elliptic IIR strainer with Blackman of FIR filter demonstrated superior consequences in SNR besides power spectral density presentation metrics than the conventional FIR filter [22]. Consequently, to remove various sounds from ECG data, we developed a cascaded FIR/IIR filter [23, 24].

## 4. Validation of Existing Filter Designs

### 4.1. IIR Filter Design

Kumari and Singh [25] have designed the two-stage IIR filter using band-pass and band-stop filters. The performance of several techniques based on FIR and IIR filter designs has been examined by them. The collected speech signal is typically coarser and requires front-end filtering. The FIR/IIR filter is widely used. It was the goal of this publication to validate the previously published Kumari and Singh [25] IIR filter design for improving speech signals.

The IIR filter is designed in two stages as combination of the band-pass and band-stop filters. The transfer function of the two-stage IIR filter design is given as follows:

(1) $$\begin{array}{c} h_{1}=\frac{0.02426s^{16}+0.2165s^{15}+1.039s^{14}+3.401s^{13}+8.38s^{12}+16.32s^{11}+25.868s^{10}+33.89s^{9}+37.05s^{8}+33.89s^{7}+25.86s^{6}+16.32s^{5}+8.38s^{4}+3.401s^{3}+1.039s^{2}+0.2165s+0.02426}{s^{16}+5.194s^{15}+13.43s^{14}+23.61s^{13}+32.38s^{12}+36.66s^{11}+34.85s^{10}+28.07s^{9}+19.36s^{8}+11.44s^{7}+5.75s^{6}+2.427s^{5}+0.8482s^{4}+0.2382s^{3}+0.05069s^{2}+0.007401s+0.0005974}. \end{array}$$

It is clear from Figure 1 that IIR filter can remove the noise at the front end for speech signal but need to carefully define the cut-off frequencies and also need improvement [10, 26].

### 4.2. Comparison of the Transfer Functions

The band-pass filters of the selected cut-off frequencies having transfer function, as an example, for ECG signal from 106 MIT-BIH data, are defined as follows:

(2) $$\begin{array}{c} h_{1}=\frac{\;0.2066{\text{s}}^{4}-0.4131{\text{s}}^{2}+0.2066}{{\text{s}}^{4}+0.5488{\text{s}}^{3}+0.4535{\text{s}}^{2}+0.1763\text{s}+0.1958}, \end{array}$$

where *h*_2_ is the band-stop filter's transfer function. A sample transfer function for ECG signal from 106 MIT-BIH data is as follows:

(3) $$\begin{array}{c} h_{2}=\frac{\begin{array}{c} 0.3201{\text{s}}^{16}+4.517{\text{s}}^{15}+30.45{\text{s}}^{14}+130{\text{s}}^{13}+393.2{\text{s}}^{12}+\\ 892.9{\text{s}}^{11}+1574{\text{s}}^{10}+2196{\text{s}}^{9}+2452{\text{s}}^{8}+2196{\text{s}}^{7}+1574{\text{s}}^{6}\\ +892.9{\text{s}}^{5}+393.2{\text{s}}^{4}+130{\text{s}}^{3}+30.45{\text{s}}^{2}+4.517\text{s }+0.3201 \end{array}}{\begin{array}{c} {\text{s}}^{16}+12.12{\text{s}}^{15}+70.25{\text{s}}^{14}+258.1{\text{s}}^{13}+672.2{\text{s}}^{12}\\ +1316{\text{s}}^{11}+2004{\text{s}}^{10}+2419{\text{s}}^{9}+2340{\text{s}}^{8}+1819{\text{s}}^{7}+113{\text{s}}^{6}\\ +559.4{\text{s}}^{5}+214.8{\text{s}}^{4}+62{\text{s}}^{3}+12.7{\text{s}}^{2}+1.649\text{s}+0.102 \end{array}}. \end{array}$$

In the further sections of the manuscript, the performance of the proposed filter is evaluated using the transfer functions [27].

### 4.3. Results of the Optimum Reduced-Order Filter Proposal

This is observed via equations (2) and (3) above, the basic IIR filter entails a 16-order, advanced-order filter. To minimize the order of the transfer function, Min-Max optimization is projected in this study. The IIR filter's numerator and denominator coefficient vectors [*b*_1_, *a*_1_] optimize Min-Max optimization. As seen in the sequential process for Min-Max optimization, transfer function coefficients are optimized consecutively. This IIR filter is termed as optimum reduced IIR (ORIIR).

### 4.4. Transfer Function Analysis of ORIIR

In this section, Table 1 represents the transfer functions aimed at several phases of the proposed lower mandate IIR filter strategy for ECG signals. As can be seen, our solution considerably reduces the filter order while also preserving the behaviour of the ECG signal, as beforehand mentioned. It is also seen that the IIR filter has a 16-order design, but after optimization, the reduced-order filter has a 2-order enterprise.

### 4.5. Design Parameters and Impacts

The FIR filter outperforms the IIR filter in terms of frequency stability. Since the zeroes in the FIR filter transfer function are fixed, this is the case. As a result, addressing the issue of IIR filter stability is a challenging task. Therefore, this manuscript is focused to analyse the stability performance.

The channel simulator's input parameters are divided into two groups. The main benefit of this filter design is that it reduces compute delay and filter order. The stability of the best reduced-order filter for transfer functions is investigated. Filters are used to minimise the effects of ECG readings on the patient's movement. In addition to filter stability, the step, impulse, and pole-zero responses are also being studied.

In this study, the evaluation of filter performance is based on the examination of transfer function (TF) stability and pole-zero plots.

Many digital filters have been designed to reduce external and internal noises. Because the digital filters are programmable, their characteristics can be modified easily, while the hardware remains the same. Digital filters can be reprogrammed to change their characteristics without needing to change the hardware. Digital filters appear to be more consistent over time than analogue filters.

#### 4.5.1. Stability and Response Analysis

The outcomes of the filtered signal response are evaluated in this part using the IIR filter's recommended design. An IIR filter is composed of a band-pass filter and a band-stop filter, and the best reduced-order filter is examined for stability and transfer properties. To eliminate noise aberrations, ECG readings are filtered. For filter stability testing, the step, impulse, and pole-zero responses are evaluated for the three filter architectures including Pan–Tompkins 32-order FIR, 60-order FIR filter, and the projected IIR filter with abridged order. Zero plots are used to measure the performance of filters based on the stability and poles of transfer functions. The amplitude besides frequency reactions of the recommended IIR filter strategy are compared first in this section.

The presentation of the FIR filter used in the Pan–Tompkins method is compared to our proposed optimum reduced IIR filter design architecture, which employs a 16th-order IIR filter. The suggested filter has a substantially higher and steadier response, allowing it to efficiently minimize signal noise.

*(1) 60-Order FIR Filter Step Responses*. This study looks at the effectiveness of a 60-order filter for a design with a cut-off frequency of *W*_*n*_ = 0.2 and band-pass ripples of 1.5 decibels (dB's). A 60-order filter is used to filter at 50 Hz. A band-pass filter is also applied to ECG signals. The 60-order filter produced in this study has a transfer function of h notch, which stands for eighth-order filter [29].

(4) $$\begin{array}{c} h_{60}=-4.168e-19s^{60}+0.0004528s^{59}0.0008864s^{58}+0.001208s^{57}-0.00127s^{56}+0.0009014s^{55}-5.451e-18s^{54}-0.001371s^{53}+0.002909s^{52}-0.004086s^{51}+0.004272s^{50}-0.002955s^{49}+3.791e-17s^{48}+0.004159s^{47}-0.008473s^{46}+0.01146s^{45}\;-0.01158s^{44}+0.00778s^{43}-2.215e-17s^{42}-0.01052s^{41}+0.02122s^{40}-0.02865s^{39}+0.02921s^{38}-0.02005s^{37}+2.962e-17s^{36}+0.02986s^{35}-0.06616s^{34}+0.1037s^{33}-0.1364s^{32}+0.1587s^{31}+0.8331s^{30}+0.1587s^{29}-0.1364s^{28}+0.1037s^{27}-0.06616s^{26}+0.02986s^{25}+2.962e-17s^{24}-0.02005s^{23}+0.02921s^{22}-0.02865s^{21}+0.02122s^{20}-0.01052s^{19}-2.215e-17s^{18}+0.00778s^{17}-0.01158s^{16}+0.01146s^{15}-0.008473s^{14}+0.004159s^{13}+3.791e-17s^{12}-0.002955s^{11}+0.004272s^{10}-0.004086s^{9}+0.002909s^{8}-0.001371s^{7}-5.451e-18s^{6}+0.0009014s^{5}-0.00127s^{4}+0.001208s^{3}-0.0008864s^{2}+0.0004528s-4.168e-19. \end{array}$$

The transfer function of Pan–Tompkins 32-order filter is as follows:

(5) $$\begin{array}{c} h_{\text{Pan\_Tomp}}=\frac{0.03125s^{12}-0.0625s^{6}+0.03125}{s^{2}–2s+1}. \end{array}$$

A mix between a band-pass and a band-stop filter, the IIR filter is a hybrid. The transfer functions for an ECG artefact reduction approach [13, 27]. It can be observed that the designed two-stage IIR filter has the transfer function of the order 16. The designed transfer function approximation used for the recent two-stage IIR filter is as follows:

(6) $$\begin{array}{c} h_{IIR}=\frac{\begin{array}{c} 0.32s^{16}+4.517s^{15}+30.45s^{14}+130s^{13}+393.2s^{12}+\\ 892.9s^{11}+1574s^{10}+2196s^{9}+2452s^{8}+2196s^{7}+1574s^{6}\\ +\;892.9s^{5}+393.2s^{4}+130s^{3}+30.45s^{2}+4.517s+0.320 \end{array}}{\begin{array}{c} s^{16}+12.12s^{15}+70.25s^{14}+258.1s^{13}+672.2s^{12}\\ +1316s^{11}+2004s^{10}+2419s^{9}+2340s^{8}+1819s^{7}+113s^{6}\\ +559.4s^{5}+214.8s^{4}+62s^{3}+12.7s^{2}+1.649s+0.102 \end{array}}. \end{array}$$

Figure 2 compared the 32-order Pan–Tompkins filter, 60-order filter, and the two-stage IIR filter magnitude responses. It can be concluded from Figure 2 that the IIR filter with two stages the better magnitude responses [28]. The basic filter used by the standard Pan–Tompkins algorithm was of 32 orders. It has many ripples in magnitude response. It justifies the hardware complexity. The modified 60-order filter as used has the reduced magnitude [30]. The overall comparison justified the effectiveness of the proposed filter response. Nevertheless, it is also required to further minimise the filter order from 16.

Figure 3 represents the comparison of three stages of our proposed optimum abridged IIR filter design for magnitude response. It is clear from Figure 3 that abridged-order filter has less magnitude response and thus may lead to amplification but has better filter response. The frequency bands that the filter will pass or reject can be used to describe the magnitude response of the filter.

This is clearly observed from Figure 3 magnitude responses that the proposed reduced-order IIR filter has the slope, which is same as magnitude response reduces to around −2 dB to −12 dB for the frequency range of 0 to 1 normalized range, while this is clear from Figure 3(b) that simple digital IIR filter although having flat response but over's the sharp cut-off in magnitude of around −40 dB at the 0.8 normalized range or (80%) frequency spectrum. Therefore, over the entire optimum reduced-order filter relatively has flat response. These data ranges are mentioned within the red colour rectangles in Figure 3.

#### 4.5.2. Group Delay Response

“Group delay” is nothing more than the lag between an input burst and its amplitude envelope in an output burst. The term “group delay” refers to the time it takes for a signal's envelope to travel through a filter.  Figure 4 represents the comparison of the group delay responses.  Figure 4(a) shows that the 60-order FIR filter has a nonlinear group delay and a varying response.

It can be clearly served from Figure 4 that optimum IIR reduced-order filter has the flat group delay response as compared to the 60-order FIR filters. A flat group delay filter's main advantage is that binary digits related to distortions are reduced. This is due to the fact that the transmitted pulses' harmonic components will all pass through the filter at the same time.

However, a magnitude response curve only conveys half the story. In addition, the phase response of filters must be considered. The phase response (the group delay response) impacts the transient response of filters [19]. Linear phase implies a flat group delay across a given bandwidth [8]. The flat group delay signifies that the filter follows the shape of the signal. In research work, Ref. [19] has presented the group delay lineation method. To justify the group delay response, the comparison of the group delay for band-pass, IIR filter, and optimum reduced-order IIR filters are evaluated.  Figure 5 has presented the comparison of the group delay for IIR filter and the reduced-order IIR filter. It is clear that significant reduction is observed in the group delay by proposed optimum reduced-order IIR filter. There is a near-linear response. The genuine character of the ECG signal should be preserved better as a result of this.

The improvement in the group delay of the filter transfer functions is clearly observed from Table 2. The quantitative performance for Mean delay, Max delay, and Min delay is presented in Table 2. The delay for band-pass filter (BPF), IIR filter, and reduced-order IIR (ROIIR) is presented in the Table 2.

To further graphically present the GD response, the peak-to-peak group delay is plotted in Figure 6. The improvement in the PP-GD values of the group delay responses is clear from Figure 6.

#### 4.5.3. Step Response of Filters

This section uses filter transfer functions to demonstrate the step response comparison for reduced-order filter design. In this study, this has proposed to optimise the IIR filter, the Min-Max optimization is applied across the coefficients of the IIR filters. The reduced-order IIR filter constructed as the transfer function of a second-order filter with step response is shown in Figure 7

(7) $$\begin{array}{c} H_{opt}\left(s\right)=\frac{3s+14}{41}. \end{array}$$

The nonlinear impulse response comparisons of the filters are presented in Figure 8. The ECG signal is analysed using the fitter application in this publication. However, the filter can be applied to a variety of other indicators as well.

It is observed from impulse response comparison form Figure 8 that reduced-order filter has less peak amplitude than 60-order filter. Moreover, we have only two impulses and nonlinear responses.

*(1) Significance of Impulse Response*. ECG signals are usually of less amplitudes of around 1 or less. Thus, it has become essential to filter the noise at the front end of ECG signal processing since most of ECG processing is implemented using on board tiny hardware. Thus, it is good enough to design the reduced-order efficient ECG filters. Thus, a reduced-order filter is favoured since it provides a lower number of impulses in the response. Reduced impulses and magnitudes are required for a step reaction. The tabular magnitude comparison of the step response and comparison with validation of the Jain and Rathore 2021 [20] is given in Table 3.

It is clear from Table 3 that our projected ROIIR filter is better suited for the real-time implementation of the filter with less step magnitude. Peak-to-peak magnitudes for step responses for IIR filters are shown in Figure 9.

### 4.6. Stability-Based Analysis

In this section, the stability requirement for various designed transfer functions (TFs) was investigated. The poles and zeroes are plotted for evaluating the stability of the specified filter responses.

#### 4.6.1. Stability Analysis

The pole-zero analysis is used to assess the stability of the 60-order filter, IIR filter, and proposed optimum reduced-order IIR filter's designed transfer functions.  Figure 10 depicts the filtered signal results and the corresponding pole zero graphs. The results of the noisy and artefact ECG channel CH-101 are compared. The ECG data help with the synthetic random noise, and the results in each row correlate with the IIR and reduced-order filters, respectively. The position of the transfer functions' poles and zeros in the z plane with respect to the unit circle determines the filter's stability. The poles must be on the left side of the z plane for the filter to be stable.

Figure 10 shows the pole-zero charts for three alternative filter designs to investigate stability difficulties and consequences. The pole and zero locations are utilised to determine the stability. It is clear from the figure that all three filters have the poles within the unit circle or on the origin. Pan–Tompkins filter has widespread poles and zeros within the unit circle. Thus, it is a case of *not stable* filter design.

For the reduced-order IIR filter, all poles and zeros lie in the origin; thus, this is the most stable case of the all. However, the proposed filter has amplitude of two poles that is greater than 1, which could lead to instability if it is not carefully built.

#### 4.6.2. Evaluation Noise Power Spectrum

The comparison of the noise power spectrum for the 60-order filter and the proposed filter design is given in Figure 11. It can be observed from Figure 11 that our designed optimum reduced-order filter offers less noise spectrum performance. However, there may be scope of improvement further.

#### 4.6.3. Phase Delay Performance

The phase delay (PD) rather than the group delay (GD) is used to determine the delay performance of a wave of a given frequency *w*. The phase delay (PD) and group delay (GD) in nonlinear phase IIR filters are typically not the same because of system's nonlinearity. It is required to design the filter with as close to linearity in order to maintain the shape of the ECG signals as shown in Figure 12.

(8) $$\begin{array}{c} \text{Ps}=360*\frac{td}{p}. \end{array}$$

Ps is the mathematical formula for phase shift, where Ps denotes the degree of phase shift, *td* denotes the time difference between signals and waves, and *p* is the wave period.

It is clear from the above figure that the suggested system achieves a nearly linear phase response. In addition, our lower order filter greatly reduces the amount of the phase delay. The justification of the improvement in the phase delay is evidently pragmatic from the judgement of the PD response for the IIR filter and ROIIR filter. The proposed ROIIR filter provides the almost flat linear phase response and thus offers better true nature of ECG signals as shown in Figure 13. The comparison of the filtered signal for the IIR filter and the reduced-order IIR filter is presented in Figure 14. This graph supports the claim that the proposed filter preserves the true nature of the ECG signal more effectively than the current filter. Phase delay and group delay responses are almost linear with the suggested filter.

### 4.7. Component Utilization Cost Summary for Filters

In this section, we have presented cost summary for the 60-order filter, the Pan–Tompkins filter, and the optimum reduced-order IIR filter as shown in Figure 15.

The comparison of the adders, multiples, and number of states used in the filter design is presented in tabular form in this section, as shown in Table 4.

It has been demonstrated that using a reduced-order filter design can significantly reduce implementation costs, allowing it to be used in on-chip applications for low latency and real-time systems. The main reason of shifting from the Pan–Tompkins filter to reduced-order filter is to make it stable and low cost.

*(1) Cost Justification*. The cost of implementation does not mean to only financial aspects, but it incorporates a number of components as adders, multipliers, and delay elements required to design the filters. Yadav et al. [24] have presented the performance evaluations of the cost implementation of different filters. Their best performance is found with elliptical filter, and the performance comparison is shown in Table 5 for the proposed IIR filter.

It can be concluded from Table 5 that proposed ROIIR filter minimized the cost of the implementation significantly.

## 5. Conclusion

This manuscript has presented the strategy results of concentrated optimum-order filter design projected at the front-end processing of the ECG signals. The first validated the filter design by Kumari and Singh [25] who have designed the two-stage IIR filter for the speech signal demising for digital hearing ads. In the current research, the similar two-stage modified IIR filter is used in context to ECG signal filtering.

Then, the results of the 60-order FIR sieve are validated for the ECG peak recognition followed by the validation of the Pan–Tompkins filter for peak detection. The prime goal of the research is to design the filter with the simple and cost-effective manner; nevertheless, it must retain the true ECG nature. In order to justify the effectiveness of the designed filter, the transfer functions are evaluated for the step response and stability analysis. The pole-zero analysis is used to assess the stability of three different filters used for ECG peak detections. It is found that proposed reduced-order filter is stable and has less impulse response magnitudes. The phase responses of the group delay of the 60-order FIR filter, the Pan–Tompkins filter, and the proposed reduced-order IIR filter are compared. It is clear from results that peak-to-peak delay and phase are minimized using the proposed IIR filter design.

Overall, it is concluded that the proposed reduced-order filter is capable of efficiently preprocess the ECG signal and used for the ECG artefact detection.

## Figures and Tables

**Figure 1:** Representing the validation and the comparison of the speech signal filtering performance FIR vs. IIR by the Prerna and Singh [25].

**Figure 2:** Comparison of the magnitude response of the three filter methodologies: (a) the Pan–Tompkins 32-order FIR filter. (b) the 60-order FIR filter from base code. (c) Our proposed IIR filter with band-pass to band-stop combination.

**Figure 3:** Magnitude response comparisons of stages of proposed reduced-order IIR filter. (a) Magnitude response of band-pass filter. (b) Magnitude response of IIR filter. (c) Magnitude response of reduced-order optimum IIR filter.

**Figure 4:** IIR filter stage step response for ECG channel filtering. (a) 60-order FIR filter group delay. (b) Pan–Tompkins filter group delay response. (c) Reduced-order IIR filter.

**Figure 5:** Comparison of group delay for IIR and reduced-order filters for ECG data filtering.

**Figure 6:** Improvement in the PP-GD values of the group delay responses.

**Figure 7:** Assessments of the step response of the proposed reduced-order IIR filter designs for the ECG filtering. (a) Step response of the Pan–Tompkins low-pass filter. (b) Step response of the 60-order FIR filter. (c) Step response of the reduced-order IIR filter.

**Figure 8:** Assessments of the step response of reduced-order filter designs. (a) Impulse response of the Pan–Tompkins low-pass filter. (b) Impulse response of the 60-order FIR filter. (c) Impulse response of the reduced-order IIR filter.

**Figure 9:** Assessment of the peak-to-peak magnitudes for step responses for IIR filters.

**Figure 10:** The stability of three different filter designs was investigated using pole-zero graphs. (a) For the Pan–Tomkins LPF filter. (b) For the 60-order FIR filter. (c) With optimum reduced-order IIR filter.

**Figure 11:** Assessment of the noise power spectrum of the proposed optimum reduced-order IIR filter design. (a) Noise power spectrum for the 60-order filter. (b) Noise power spectrum of the proposed reduced-order filter.

**Figure 12:** The performance comparisons of the offered phase delay by the IIR filter designs. (a) Phase delay of the 60-order FIR filter design. (b) Phase delay of the optimum reduced-order IIR filter design.

**Figure 13:** Filtered signal to justify the nature of the ECG signal. (a) Filtered signal plots. (b) Zoomed IIR filtered signals. (c) Zoomed reduced-order IIR filtered signals.

**Figure 14:** Comparison of the phase delay (PD) of IIR filter and reduced-order IIR filter.

**Figure 15:** The cost implementation of filters. (a) Cost for the 60-order filter. (b) Cost for the Pan–Tompkins filter. (c) Cost of the optimization-based optimum reduced-order filter.

**Table 1:** Comparison of transfer functions for various filters used in ECG peak detection using the filter design.

Filter technique	Considered transfer functions
FIR 60-order LPF (low-pass filter)	*h*_60_ = −4.168*e* − 19 *s*^60 + 0.0004528 *s*^59 0.0008864 *s*^58 + 0.001208 *s*^57 − 0.00127 *s*^56 + 0.0009014 *s*^55 − 5.451*e* − 18 *s*^54 − 0.001371 *s*^53 + 0.002909 *s*^52 − 0.004086 *s*^51 + 0.004272 *s*^50 − 0.002955 *s*^49 + 3.791*e* − 17 *s*^48 + 0.004159 *s*^47 − 0.008473 *s*^46 + 0.01146 *s*^45 − 0.01158 *s*^44 + 0.00778 *s*^43 − 2.215*e* − 17 *s*^42 − 0.01052 *s*^41 + 0.02122 *s*^40 − 0.02865 *s*^39 + 0.02921 *s*^38 − 0.02005 *s*^37 + 2.962*e* − 17 *s*^36 + 0.02986 *s*^35 − 0.06616 *s*^34 + 0.1037 *s*^33 − 0.1364 *s*^32 + 0.1587 *s*^31 + 0.8331 *s*^30 + 0.1587 *s*^29 − 0.1364 *s*^28 + 0.1037 *s*^27 − 0.06616 *s*^26 + 0.02986 *s*^25 + 2.962*e* − 17 *s*^24 − 0.02005 *s*^23 + 0.02921 *s*^22 − 0.02862 *s*^21 + 0.02122 *s*^20 − 0.01052 *s*^19 − 2.215*e* − 17 *s*^18 + 0.00758 *s*^17 − 0.01158 *s*^16 + 0.01146 *s*^15 − 0.008473 *s*^14 + 0.004159 *s*^13 + 3.791*e* − 17 *s*^12 − 0.002955 *s*^11 + 0.004272 *s*^10 − 0.004086 *s*^9 + 0.002909 *s*^8 − 0.001371 *s*^7 − 5.451*e* − 18 *s*^6 + 0.0009014 *s*^5 − 0.00127 *s*^4 + 0.001208 *s*^3 − 0.0008864 *s*^2 + 0.0004528 *s* − 4.168*e* − 19 [28]

Pan–Tompkins 32-order LPF	*h*_32_=(0.03125*s*^12^ − 0.0625*s*^6^+0.03125)/(*s*^2^ − 2*s*+1)
BPF (band-pass filter)	*h*_1_=(0.2066*s*^4^ − 0.4131*s*^2^+0.2066)/(*s*^4^+0.5488*s*^3^+0.4535*s*^2^+0.1763*s*+0.1958)
16-order IIR filter	$\begin{array}{c} h_{2}=\left(0.32s^{16}+4.517s^{15}+30.45s^{14}+130s^{13}+393.2s^{12}+892.9s^{11}+1574s^{10}+2196s^{9}+2452s^{8}+2196s^{7}+1574s^{6}+\;892.9\;s^{5}\;+393.2\;s^{4}+130\;s^{3}+30.45\;s^{2}+4.517\;s\;+\;0.320\right)\\ s^{16}+12.12s^{15}+70.25s^{14}+258.1s^{13}+672.2s^{12}+1316s^{11}+2004s^{10}+2419s^{9}+2340s^{8}+1819s^{7}+113s^{6}+559.4s^{5}+214.8s^{4}+62s^{3}+12.7s^{2}+1.649s+0.102/ \end{array}$

Optimum reduced-order IIR filter	*h*_*opt*_=(3*s*+14)/41

**Table 2:** Quantitative performance of the group delay.

Parameter	BPF	IIR	ROIIR
Mean GD	−1.37*E* − 04	2.03*E* − 05	−0.015
Max GD	0.9	1.9867	−4.66*E* − 04
Min GD	−2.3979	−0.4538	−0.2142
Peak to Peak Swing	3.2979	2.4405	**0.213734**

**Table 3:** Magnitude performance evaluation of impulse response with the IIR filter.

Magnitude	Jain [20] ROIIR	IIR ECG filter	ROIIR ECG filter
Min Magnitude	0.423	0.8331	0.34146
Max Magnitude	0	−0.136	0.02041
Peak to Peak	0.42	0.9961	0.32105

**Table 4:** A comparison of design implementation costs for filters.

Cost parameters	60-order	Pan–Tompkins	Proposed optimum reduced-order filter
Number of used multipliers	35	4	3
Number of used adders	34	4	1
Number of states	34	12	1
Multiplications required per input signals	35	4	3
Additions required per input signals	34	4	1
Numerator length	36	13	2
Denominator Length	1	3	1
Stability	No	Yes	Yes

**Table 5:** Cost implementation justification comparison.

Cost parameters	Yadav et al. [26]	Proposed ROIIR
Number of used multipliers	32	3
Number of used adders	32	1
Order of filter	8	2
Stable	Yes	Yes

## Data Availability

The data underlying this article are derived from online sources in the public domain as PhysioNet. The heart rates (ECG) are measured over 3 R-R intervals in beats per minute and available at https://physionet.org/physiobank/database/html/mitdbdir/records.htm.
